# miR-16 and Fluoxetine Both Reverse Autophagic and Apoptotic Change in Chronic Unpredictable Mild Stress Model Rats

This article has been retracted.

**DOI:** 10.3389/fnins.2017.00428

**Published:** 2017-07-25

**Authors:** Yang Yang, Zhiying Hu, Xiaoxue Du, Henry Davies, Xue Huo, Marong Fang

**Affiliations:** ^1^Institute of Neuroscience, Zhejiang University School of Medicine Hangzhou, China; ^2^Department of Obstetrics and Gynecology, Hangzhou Red Cross Hospital Hangzhou, China

**Keywords:** depression, miR-16, fluoxetine, autophagy, apoptosis, 5-HT2a

## Abstract

In the clinic selective serotonin reuptake inhibitors (SSRIs), like Fluoxetine, remain the primary treatment for major depression. It has been suggested that miR-16 regulates serotonin transporters (SERT) via raphe nuclei and hippocampal responses to antidepressants. However, the underlying mechanism and regulatory pathways are still obtuse. Here, a chronic unpredicted mild stress (CUMS) depression model in rats was established, and then raphe nuclei miR-16 and intragastric Fluoxetine injections were administered for a duration of 3 weeks. An open field test and sucrose preference quantification displayed a significant decrease in the CUMS groups when compare to the control groups, however these changes were attenuated by both miR-16 and Fluoxetine treatments. A dual-luciferase reporter assay system verified that hsa-miR-16 inhibitory effects involve the targeting of 3′UTR on the 5-HTT gene. Expression levels of miR-16 and BDNF in the hippocampus were examined with RT-PCR, and it was found that increased 5-HT2a receptor expression induced by CUMS can be decreased by miR-16 and Fluoxetine administration. Immunofluorescence showed that expression levels of neuron NeuN and MAP-2 in CUMS rats were lower. Apoptosis and autophagy levels were evaluated separately through relative expression of Bcl-2, Caspase-3, Beclin-1, and LC3II. Furthermore, CUMS was found to decrease levels of hippocampal mTOR, PI3K, and AKT. These findings indicate that apoptosis and autophagy related pathways could be involved in the effectiveness of antidepressants, in which miR-16 participates in the regulation of, and is likely to help integrate rapid therapeutic strategies to alleviate depression clinically. These findings indicate that miR-16 participates in the regulation of apoptosis and autophagy and could account for some part of the therapeutic effect of SSRIs. This discovery has the potential to further the understanding of SSRIs and accelerate the development of new treatments for depression.

## Introduction

Major Depressive Disorder (MDD) is characterized by a pervasive and persistent low mood, which is affecting nearly 300 million people worldwide, with the prevalence of depression standing at around 19% of the population. Statistical information from the World Health Organization (WHO) indicates that by 2030 depression will be the greatest source of disability worldwide (Albert and Francois, 2010; Albert and Fiori, 2014). It is true that a large number of antidepressant drugs are already available for depressive disorders treatment. However, the majority of these drugs have certain disadvantages, such as delayed efficacy and numerous side effects (Kaufmann et al., 2016). Previous reports have revealed that ~30% of patients do not benefit from drug therapy. The lack of understanding of SSRI mechanism is exemplified by the fact that to date it is still not understood why, despite brain levels of serotonin increasing just hours after administration, a perceived antidepressant effect by the patient takes weeks. Therefore, it is still necessary to do further studies that focus on the mechanisms underlying depression in order to seek more efficient clinical treatments (Bortolozzi et al., 2014; Xu et al., 2016).

Serotonin (5-hydroxytryptamine, 5-HT) is a monoamine neurotransmitter and is mainly found in blood platelets and in the central nervous system (CNS) in animals and humans. It is widely considered to be a contributor to feelings of well-being and happiness (Ertugrul et al., 2007). Serotonin plays an important role in psychiatric disorders like depression, anxiety and Parkinson's disease. The serotonin hypothesis for depression was put forward in the 1960s, suggesting 5-HT deficiency in the brain contributes to the onset of depression. Until now, selective 5-HT reuptake inhibitors (SSRIs), like Fluoxetine, remain the most crucial antidepressant treatment (Rayen et al., 2011). Pandey and her colleagues have shown that 5-HT2A receptor modulation is associated with depressive-like behavior. Depressive-like behaviors can be significantly reversed by applying treatment with the 5-HT2A receptor antagonist BIP-1 combined with the antidepressant amitriptyline (Pandey et al., 2010). Zaniewska et al. demonstrated that the acute 5-HT2A receptor antagonist M100907 can reduce antidepressant like effects, similar to antidepressant drugs (Zaniewska et al., 2010).

Micro ribonucleic acids (miRNA) are a subclass of about 22 nucleotide (nt) noncoding RNA species, which function primarily by disrupting target messenger RNA (mRNA) expression. O'Connor et al. revealed that miRNAs play a regulatory role during neuronal development, neurogenesis and synaptic plasticity, which are all crucial processes in the CNS and any undermining activities to these processes can be involved in the development of depression (O'Connor et al., 2012). More specifically, Katelin F. Hansen suggested that miRNAs show remarkable potential in the treatment of clinical depression and some other mood disorders (Hansen and Obrietan, 2013; O'Connor et al., 2013). Previous studies have demonstrated that miR-16 is involved in brain development, function and diseases including depression. In the study of Baudry et al. it was proposed that miR-16 contributes to the therapeutic action of SSRI antidepressants in monoaminergic neurons (Baudry et al., 2010). Previous research has proved that chronic administration of the SSRI fluoxetine in mice leads to an increased level of miR-16 expression in serotonergic raphe nuclei, leading to a reduction in SERT. Moreover, during early life, depressive behavior induced by stress is connected with abnormal expression levels of BDNF and miR-16 in the hippocampal region (Bai et al., 2012).

In this present study, a CUMS model, which is considered to be the most representative of depression in humans, was employed in order to explore miRNA function on stress related dysregulation. miRNAs are highly conserved among mammals, therefore study results can be well applied to humans, and thus beneficial for the development of clinical drugs (Zurawek et al., 2016). Recently, the potential role of regulatory apoptosis and autophagy in neurodegenerative diseases and tumor suppression has been widely investigated (Polajnar and Zerovnik, 2014). It has been hypothesized that neurodegenerative diseases such as depression, Parkinson's and Alzheimer's could result from excessive autophagy and apoptosis. Previous research has revealed that autophagy is upregulated swiftly in ischemia and upregulated gradually in chronic diseases like depression, but the actual mechanisms underlying apoptosis-autophagy interactions in depression remain unclear (Li et al., 2015; Yang et al., 2015).

Another important angle for neurodegenerative disease study could be signal transduction pathways, which promote cellular survival and proliferation via effects on cellular metabolism. It has been shown that activation of the phosphoinositide-3-kinase/serine-threonine kinase Akt/mammalian target of rapamycin (PI3K/Akt/mTOR) pathway could have very crucial effects on cell proliferation and apoptosis of cells involved in brain function (Tessier et al., 2015). Weiwei Tao et al showed that Liquiritigenin could alleviate depressive-like symptoms induced by CUMS, and this protective role might be conducted through regulating PI3K/Akt/mTOR mediated BDNF/TrkB pathway in CUMS mice hippocampus (Tao et al., 2016). Our previous study showed that cerebral ischemic injury may inactivate PI3K/Akt/mTOR pathways. Considering the neuroprotective role of the PI3K/Akt/mTOR pathway in previous studies and combining evidence from other depression studies, we hypothesized that, like Fluoxetine, miR-16 may also be able to alleviate depressive symptoms through the up-regulation of PI3K/Akt/mTOR pathways and the reduction of both apoptosis and autophagy.

## Materials and methods

### Ethics statement

This study was performed following the Guide for Care and Use of Laboratory Animals and was approved by the Laboratory Animal Center of Zhejiang University. All experiments were conducted in accordance with the guidelines from the Anatomy Lab in the School of Basic Medical Sciences, Zhejiang University.

### Animal preparation

Sprague-Dawley rats weighing 250–280 g were provided by the Laboratory Animal Center of Zhejiang University. In order to minimize the number of experimental animals, best possible care was provided. All the animals used in this study were pathogen-free, kept under a 12 h light/dark cycle in separated clean cages in an air-conditioned room with a constant temperature of 24 ± 1°C. In this study, all rats had free access to food and water and all feeding procedures were approved by the Ethics Committee for Use of Experimental Animals in Zhejiang University. The animals were first kept in group before experiments, and then housed individually during the CUMS process. Since the CUMS started, the animals were single housed throughout the entire experiments. All the operations were in accordance with the National Institutes of Health (NIH) Guide for the Care and Use of Laboratory Animals guidelines.

### Experimental groups

All the animals were first subjected to behavioral tests before and after CUMS. The total 96 rats used afterwards were selected as the successful model rats. Then separate the rats to 8 groups, each with 12 animals. Upon sacrificing, 6 of the rats from each group for fresh tissue extraction (protein and RNA extractions), another half for perfusion and fixed with 4% paraformaldehyde (histology analysis). Brain tissues were removed after sacrifice for RNA and protein extraction. The experimental groups were as follows: (1) Control1 group (Cont1), which were sacrificed after 4 weeks, (2) CUMS1 group, which received a 4 week stress treatment, (3) Vector group, which were injected with vectors after 4 weeks of stress treatment, (4) miR-16 group, which were injected with an miR-16 lentivirus after 4 weeks of stress treatment, (5) Control2 group(Cont2), which were sacrificed after 7 weeks, (6) CUMS2 group, which received 4 weeks of stress treatment, but were then kept alive for an additional 3 weeks before being sacrificed, (7) Vehicle group, which were treated for 3 weeks with a vehicle after an initial 4 weeks of stress treatment, (8) Fluoxetine group, which were given 3 weeks of Fluoxetine after an initial 4 weeks of stress treatment.

### Lentivirus information and drug administration

Our targeted miR-16 fragment was inserted into a vector named pHBLV-U6-ZsGreen through EcoR I and BamH I digestion sites, and the expression was regulated by a U6 promoter. This vector contains a CMVIE promoter to have ZsGreen expression. Primers used in this process were:

hsa-miR-16-F (BamHI) GACGGATCCGCTCTAGAAATTTAAGGAAATTC; hsa-miR16-R (ECORI) GACGAATTCCTTGTTGTGATATCAAGTATATGG;

At the time point of 4 weeks into the CUMS process, the rats in the miR-16 group and vector group were ready for stereotaxic surgery. Briefly, after anesthetising with 10% chloral hydrate intraperitoneally, the viral solution and the vector only solution were bilaterally injected through a burr hole into raphe nucleus. According to the Rats' Brain Atlas, the injection coordinate was selected as anteroposterior, *Y* = 7.8 mm from bregma; mediolateral, *X* = 0 mm; dorsoventral, *Z* = 8.5 mm. The injection speed was controlled using a 1 μl syringe microinjector at a rate of 0.5 uL/min and a total volume of 2 μl. The needle was left in place for an additional 5 min afterwards. Rats were then laid down in a heated chamber to recover from anesthesia. The Fluoxetine group and the Vehicle group were given intragastric Fluoxetine (Lilly, PATHEON FRANCE and 10 mg/kg/d) and physiological saline respectively for 3 weeks after an initial 4 weeks of CUMS.

### Experimental design and CUMS procedure

The diagram in Figure 1A outlines the experimental procedure that we used in this study. At the time points of pre-CUMS, after stereotaxic injection surgery and after Fluoxitine treatment, open field tests and sucrose preference tests were performed. The CUMS period lasted for 4 weeks and, as can be seen in Figure 1B, the treatment included tail pinching for 5 min, food deprivation for 24 h, swimming at 4°C for 5 min, a tilted cage for 90 min, confined space for 90 min, soiled cage overnight, noise stress for 12 h, tail suspension for 20 min and water deprivation for 24 h. Cont1, CUMS1, Vector and miR-16 groups were sacrificed after behavior tests at the time point of 5 weeks. Cont2, CUMS2, Vehicle and Fluoxetine groups were sacrificed after behavior tests at a time point of 7 weeks.

**Figure 1:** Process diagrams for experimental procedures and daily stressful events of CUMS rat model. **(A)** Process diagram for the experimental procedure, which is in accordance with that described in the Materials and Methods Section. The behavioral tests, including the open field test and the sucrose consumption test, were measured before CUMS, after CUMS and 1 day before sacrifice. Stereotaxic injection of miR-16 and the vector were conducted 4 weeks into CUMS. Cont1, CUMS1, Vector and miR-16 groups were sacrificed 1 week after the injection. Fluoxetine treatment was given periodically after CUMS, and continued for 3 weeks. Cont2, CUMS2, Vehicle and Fluoxetine groups were sacrificed after behavioral tests. **(B)** Process diagrams of daily stressful events of CUMS rat model. Rats in each group, except for the control group, were exposed to this.

### Behavior tests

The open field test was done with VIDEOTRACK V3. The arena consisted of an open rectangular plastic box (80 × 80 × 40 cm) with 16 squares marked with red lines on the floor. All the tests were carried out between 14:00 and 17:00 in an air conditioned and, soundproofed room with no natural light source. Experiments were carried out and observed in a dark box, except for lights inside the box that used for video capturing. After VIDEOTRACK V3 was set up and linked to a computer, rats were placed individually at the center of the field and allowed to explore the area freely for 5 min. The activity of the rats was recorded by an overhanging camera, which recorded all tracks of the rats' movement. Between each rat trial, the arena was cleaned with 70% alcohol to keep it clean and avoid any infection. Total distance, rearing movements, center entries, and center distance were recorded for each rat.

Each sucrose preference test was done over 3 consecutive days. The first day (24 h) was for the rats time to become accustomed to sucrose solution for, so were housed individually with free access to two bottles of sucrose solution (1%, w/v and 100 ml). On day 2 (24 h), one bottle of sucrose solution was substituted with 100 ml of pure water. On day 3, the rats were tested after 23 h of complete water and food deprivation. For the test the rats were given free access to two bottles [100 ml of sucrose solution (1%, w/v) and 100 ml of pure water]. The solution weights were recorded at the beginning and the end of the 1 h test and sucrose preference rate was calculated according to the formula: Sucrose preference rate = sucrose consumption/total solution consumption^*^100%. Reduction rates of sucrose preference were assumed to reflect anhedonia levels.

### *In vitro* luciferase assay

In order to elucidate the target role miRNAs on these transcripts, *in vitro* luciferase assays were performed to test miR-target interaction between the 3′ UTR of 5-HTT. The genomic sequencing of the inserted miR-16 is shown in Figure 3A. After the construction of the miR-16 (lentivirus) over-expression vector and the lentiviral 3′UTR of 5-HTT, we did co-transfection with these two plasmids to HEK293T cells to verify the efficiency of miR-16 in combination with the gene of interest. Moreover, the purpose of the dual luciferase reporter gene detection system was to verify the regulation of hsa-miR-16 on the 3′UTR of 5-HTT. Both hsa-miR-16WT and hsa-miR-16MUT were co-expressed with lentiviral of 3′UTR of 5-HTT, the luciferase expression changes were shown in **Figure 3B**.

### Immunofluorescence

Rats were anesthetized with 10% chloral hydrate and then transcardially perfused by 500 mL of 0.9% saline to flush the vascular blood and then perfeused with 4% paraformaldehyde in 0.01 M phosphate-buffered saline (PBS, pH 7.4). Brains tissues were obtained after perfusion and fixed with 4% paraformaldehyde, then on the next day tissues were transferred to 30% sucrose solution overnight before frozen sample preparation. Frozen sections, about 18 um thick, were rinsed in 0.01 M PBS for 5 min. After drying at 37°C, sections were moved to room temperature (RT) for 1 h and blocked with 5% normal goat serum. Then primary antibodies were applied in the following concentrations at 4°C overnight: 5-HT2a (Abcam, ab16028, 1:200), mTOR (EPITOMICS, p42345, 1:200), MAP-2 (17490-1-AP, 1:200), and NeuN (Abcam, ab104224, 1:1,000). As for the negative control sections, 0.01 M PBS was used to replace the primary antibody (Li et al., 2015; Yang et al., 2015). The sections were washed with 0.01 M PBST for 5 min three times on the following day, and then incubated with the secondary antibody containing FITC goat anti-rabbit IgG (1:100, Boster BA1105), Alexa Fluor® 488 and Alexa Fluor® 594 for 1 h at RT. They were then washed again three times with PBST, following PI (propidium Iodide BB-4136-100T) staining for 10 min at RT, then the sections were ready for fluorescence after the mounting medium had been added to the slides. Finally, observation and pictures were taken with a fluorescence microscope (Olympus BX51, NIKON, Japan) at excitation/emission wavelengths of 550/570 nm (Cy3, red) and 492/520 nm (FITC, Green and blue).

### Western blotting

Total proteins of the hippocampus brain tissue were extracted from each group with 1% PMSF (Phenylmethanesulfonyl fluoride, Beyotime ST505) in 1 mL of ice-cold RIPA buffer, with added protease inhibitor cocktail EDTA-free and phosphatase inhibitors. After homogenizing and centrifuging at 12,000 rpm for 20 min at 4°C, the supernatant proteins were preserved at −80°C and ready to be measured for concentration. The concentration of all samples were determined with BCA kits (KeyGEN, Nanjing, China). A total of 20 μg of protein from each sample was subjected to electrophoresis on 12% SDSPAGE gel using a constant voltage. Next, the proteins were transferred to a polyvinylidene difluoride (PVDF) membrane with the Bio-Rad TransBlot apparatus. The transfer process was conducted under 100 V of electricity for 120 min. Afterwards, the membranes were blocked to TBST containing 5% non-fat milk for 2 h at RT. And then the membranes were incubated with primary antibody overnight at 4°C. The following primary antibodies were used in this study: rabbit polyclonal antibody against β-actin (Abmart #P30002, 1:2,000), 5-HT2A (Abcam, ab16028, 1:1,000), Beclin-1 (CST#3495, 1:1,000), LC-3 (Abcam, ab #3868, 1:1,000), mTOR (EPITOMICS, p42345, 1:1,000), PI3K (Cell Signaling Technology, Inc., USA; 1:1,000), AKT (CST#2938, 1:1,000), Bcl-2 (1:1,000; Santa Cruz Biotechnology, Santa Cruz, CA, USA), and caspase-3 (CST#9665, 1:1,000). The membrane was washed with TBS containing 0.05% Tween 20 (TBST) on the following day. After washing 3 times for 5 min each, the membranes were incubated with goat antirabbit IgG antibody (AURAGENE, SA009) at room temperature for 2 h, and then washed with TBST 3 more times, also for 5 min each. Finally, membranes were ready to be exposed to Hyperfilm detection after incubating with the ECL system. The greyscale value of each band was analyzed by Quantity One program. Each experiment was done 3 times.

### Real-time PCR

Real-time PCR was conducted to detect RNA expression level of BDNF and miR-16 in hippocampal tissues. The Trizol (Invitrogen) extraction reagent, was used to extract hippocampal RNA and all procedures were carried out according to the manufacturer's instruction. Next, concentration and purity of the RNA samples were determined by Thermo NanoDrop 2000. One microgram of RNA from each sample was reverse transcripted into cDNA according to the instructions of the DBI-2220 Bestar™ qPCR RT Kit. Real-time PCR specific primers for rat miR-16, BDNF and β-actin (internal control) were designed using Primer Express software. The primers used in this study were as follows: miR-16 Forward: 5′-TAGCAGCACGTAAATTGGCG-3′;

U6 Forward: 5′-GCAAGGATGACACGCAAATTC-3′;
miR-16 and U6 common Reverse: 5′-GTGCAGGGTCCGAGGT-3′;
BDNF Forward: 5′-TGGCTGACACTTTCGAACAC-3′;
BDNF Reverse: 5′-AGAAGAGGAGGCTCCAAAGG-3′;
β-actin Forward: 5′-GGAGATTACTGCCCTGGCTCCTA-3′;
β-actin Reverse: 5′-GACTCATCGTACTCCTGCTTGCTG-3′.

Real-time PCR protocol was done following instructions from DBI-2044 Bestar® SybrGreen qPCR master mix. The reaction program for the PCR was as follows: 50°C for 2 min; 95°C for 10 min; 40 cycles of 95°C for 5 s, 55°C for 30 s, 72°C for 30 s. All mRNA expression levels were detected by RT-PCR and detailed primer information can be seen in the Materials and Methods Section. Later the results were analyzed with the Biorad CFX manager program, version 3.0. Each experiment was done 3 times.

### Statistic analysis

Cont1 and cont2 groups were served as the control vs. CUMS model groups and vector/vehicle served as the control vs. miR16/Fluoxetine group respectively for the experiment in this study. All the quantitative data in this study are presented as mean ± SD. The staining quantifications were conducted by five randomly selected fields of immuno-stained tissues in each specimen. Data were presented as the mean of 5 fields for each specimen, one of the representative image was presented in the figures accordingly. Data analysis and histograms were done with Graph Pad Prism 5. The established *t*-test was used to analyze statistical differences between two groups. Values of *P* < 0.05 were considered significant. SPSS 16.0 program was employed to determine statistical significance using a oneway analysis of variance (ANOVA) way. The null premise was discarded at the level of 0.05. Western-blot was analyzed and evaluated by Quantity One. Again, *P* < 0.05 was considered to have statistical significance.

## Results

### (Luciferase assay) hsa-miR-16 conducted its regulatory role through the 3′UTR binding site on 5-HTT

In this study, dual luciferase gene detection was conducted to verify the inhibition effect hsa-miR-16 has on its target gene 5-HTT. In order to reaffirm 3′UTR as the active site between hsa-miR-16 and its target gene 5-HTT, the expression of luciferase, which contained 3′UTR of 5-HTT, was measured under hsa-miR-16 over-expression. A 3′UTR full-length clone of 5-HTT mRNA was converted to a Renilla luciferase reporter vector, and this construction was co-transfected with wild-type miR-16 to determine if 5-HTT is one of the miR-16 target genes. The genomic information of miR16 can be seen in **Figure 3A** and a simple diagram of this experiment is shown in **Figure 3B**. The miR-16 expression construction vector was introduced into HEK 293T cells and a plasmid transfection luciferase reporter assay was done to check whether the 3′UTR sequence of 5-HTT contains the active sites for miR-16. It can be seen in [*F*_(3, 8)_ = 15.37, *P* = 0.0011, **Figure 3C**] that hsa-miR-16 can regulate Luciferase expression (*P* = 0.0077 vs. WT mimic NC, ^**^P < 0.01) with a decreased expression level. However, this regulation disappeared after a deliberate mutation to the binding site, indicating that hsa-miR-16 indeed conducts its regulatory role through this binding site and controls Luciferase expression.

### The histological verification of miR16 injection was confirmed by fluorescence microscopy

On the 7th day after miR16 injection by stereotaxic surgery, the brain tissues were harvested for fluorescence microscopy to verify the expressional location. Strong expression of miR16 in rat's raphe nuclei was confirmed immunofluorescently (Supplementary Figure 1, green), the nuclei of all the cells were stained by DAPI (Supplementary Figure 1, blue).

### miR-16 can ameliorate depressive behavioral changes caused by CUMS in a similar way to fluoxetine

The sucrose preference test: At enrollment time, there was no significant difference between any of the rats in the amount of sucrose consumption. Figure 2F [*F*_(2, 14)_ = 170.2, *P* < 0.0001] shows statistically significant differences in sucrose consumption between each group of rats. Rats in the control group were seen to show no significant change in the proportion of consumption throughout the whole testing process (*P* > 0.05). With time, the proportion of sucrose consumption decreased gradually in CUMS1, CUMS2, vector, and vehicle groups. Compared with the control group, rats in the CUMS1 and CUMS2 groups had significantly (*P* < 0.0001) less sucrose consumption. Consumption in the miR-16 (*P* < 0.0001) and Fluoxetine (*P* < 0.0001) groups were more than CUMS1 and CUMS2, but less than the controls.

**Figure 2:** Behavioral test comparison of each group immediately prior to sacrifice. Representative pictures of behavioral tests immediately prior to sacrifice show differences between each group, and selective movement tracks. The histograms show total distance **(A)**, rearing movements **(B)**, center entries **(C)**, and center distance **(D)** in each group. Values are means ± SEMs. ^*^P < 0.05; ^**^P < 0.001; ^***^P < 0.0001. **(E)** The selective movement locus from each group prior to sacrifice can be seen. **(F)** The histograms show sucrose preference in each group. Values are the means ± SEMs. ^*^P < 0.05; ^**^P < 0.001; ^***^P < 0.0001.

**Figure 3:** Hsa-miR-16 can regulate Luciferase expression by binding to the 3′UTR region of 5-HTT. The dual-luciferase reporter assay system verifies that hsa-miR-16 targets 3′UTR of gene 5-HTT and exerts an inhibitory effect. **(A)** Genome sequence of miR-16 is shown in the figure, and the highlighted part is stem-loop region. **(B)** Simple diagram of the luciferase experiment. The WT miR-16 and MUT miR-16 were co-transfected with 5-HTT. In order to reaffirm 3′UTR as the active site between hsa-miR-16 and its target gene 5-HTT, the expression of luciferase, which contained 3′UTR of 5-HTT, was measured under hsa-miR-16 over-expression. **(C)** The histogram shows that hsa-miR-16 can regulate Luciferase expression (^**^P < 0.01) via the 3′UTR region of 5-HTT, while a mutation of the binding site stops this effect, thus confirming that hsa-miR-16 regulates Luciferase expression through this binding sites.

The open field test: Representative images of tracked movements for each group can be seen in Figure 2E. In this study total distance [*F*_(7, 16)_ = 28.4, *P* < 0.0001, Figure 2A], rearing movements [*F*_(7, 16)_ = 17.32, *P* < 0.0001, Figure 2B], center entries [*F*_(7, 16)_ = 20.07, *P* < 0.0001, Figure 2C] and central distance [*F*_(7, 16)_ = 187.4, *P* < 0.0001, Figure 2D] were chosen to represent mobility capability. The activity of rats in CUMS1 and CUMS2 groups at week 4 and week 7 were lower than the control (*P* < 0.05). From Figures 2A–D it can be seen that in comparison with CUMS1 and CUMS2 groups, MiR-16 (*P* = 0.0025, 0.0106, 0.0331, 0.0031 vs. Cont1) and Fluoxetine (*P* = 0.0033, 0.0090, 0.0179, 0.0161 vs. Cont12) groups had significantly more movement. The open field test showed that the depression model was a success in that space and range were significantly reduced. Moreover, injection treatment with miR-16 lentivirus and Fluoxetine treatment achieved a certain amelioration depressive behaviors.

### MiR-16 can restore post CUMS BDNF expression levels in a similar capacity to fluoxetine

BDNF (brain derived neurotrophic factor) and miR-16 expression changed with relation to each other, so this suggests an interaction between them. Figure 4B [*F*_(7, 16)_ = 25.43, *P* < 0.0001] shows a large decrease in BDNF expression in both CUMS1 and CUMS2 in comparison to Cont1 and Cont2 (*P* = 0.0027 vs. Cont1, 0.0004 vs. Cont2). However, miR-16 and Fluoxetine treatments appear to lessen this decrease. In Figure 4A, the expression of miR-16 in the hippocampus is shown, and there is a significant decrease in miR-16 (*P* = 0.036 vs. CUMS1) and Fluoxetine (*P* = 0.0017 vs. CUMS2) groups when compared with CUMS1 and CUMS2. In the hippocampus, decreased levels of miR-16 correlate to increases in SERT, which can have an anti-depressive effect. The regulatory diagram can be seen in Figure 4C. Moreover, there was no significant change between the miR-16 group and the Fluoxetine group, which means these two protect similarly toward CUMS derived depressive symptoms and that in both cases this could be done by regulating BDNF expression via miR-16 in the hippocampus.

**Figure 4:** Hypothetical diagram of miR-16 and BDNF network regulation through autophagy and apoptosis. miR-16 and Fluoxetine treatment at the Raphe nucleus can generate autophagic and apoptotic changes in the hippocampus through regulation of BDNF. Histograms show relative expression of miR-16 **(A)** and BDNF **(B)** from RT-PCR. Values are the means ± SEMs. ^*^P < 0.05; ^**^P < 0.001; ^***^P < 0.0001. **(C)** Hypothetical diagram of how the miR-16 and BDNF networks regulate autophagy and apoptosis. Fluoxetine and miR-16 injection into the Raphe nucleus presented protective effects on CUMS derived depressive symptoms and that in both cases this is done by regulating BDNF expression via miR-16 in the hippocampus.

### miR-16 is involved in the regulation of 5-HT2a expression after CUMS

Expression change of 5-HT2a was detected by both western blotting and immunofluorescence. The representative images of western blotting and immunofluorescence can be seen in Figures 5A,C, which showed an increased expression level of 5-HT2a after CUMS when compared with control groups, while the increase can be ameliorated by both miR-16 and Fluoxetine. The increasing tendency in the CUMS groups was in agreement with an abundance of evidence that has already proved reduced 5-HT neurotransmission to be a fundamental change in depression. And miR-16 injection was as protective as Fluoxetine in the CUMS model. From both western blotting and immunofluorescence detections, which showed similar trends. The histogram from 5-HT2a staining [*F*_(7, 16)_ = 78.74, *P* < 0.0001, Figure 5B] showed that CUMS groups are increased compared to the control (*P* = 0.0005 vs. Control, ^***^P < 0.0001), whereas miR-16 and Fluoxetine (*P* = 0.0003 vs. CUMS1, *P* = 0.0014 vs. CUMS2, ^**^P < 0.01) treatment groups attenuated this increasing tendency. Optical densities of respective protein bands were presented in Figure 5D [*F*_(7, 16)_ = 15.92, *P* < 0.0001]. 5-HT2a expression levels were down-regulated in the miR-16 group (*P* = 0.0076 vs. CUMS1, *P* = 0.0348 vs. CUMS2, ^**^P < 0.01) when compared with the CUMS and vector groups, but still had more expression than the Control group (*P* = 0.0019 vs. Cont1, *P* = 0.001 vs. Cont2). Since all antidepressant treatment, including serotonin reuptake inhibitors (SSRIs) like Fluoxetine, increase 5-HT neurotransmission directly or indirectly, it can be deduced that miR-16 might improve depressive symptoms in the CUMS rat model through reducing expression levels of 5-HT2a.

**Figure 5:** 5-HT2a upregulation after CUMS was observed from Western blot and immunofluorescence staining. Representative images of 5-HT2a by immunofluorescence staining **(A)** are in accordance with western blot **(C)** analysis of protein levels of 5-HT2a and β-actin in the rat hippocampus of each group. **(B)** The histogram from 5-HT2a staining showed that CUMS groups are increased compared to the control, whereas miR-16 and Fluoxetine treatment groups attenuated this increasing tendency. Values are the means ± SEMs. ^*^P < 0.05; ^**^P < 0.001; ^***^P < 0.0001. **(D)** Optical densities of respective protein bands **(C)** were analyzed and normalized to β-actin. Results were expressed as means ± SDs from three independent experiments. From the histogram, the expression of 5-HT2a in each group has a comparatively similar fluctuation to immunochemistry staining.

### Immunofluorescence detection showed MAP-2 and NeuN expression to increase in both miR-16 and fluoxetine groups

Both MAP-2 and NeuN reflect levels of certain neuronal cells. From the representative images in Figure 6B, immunofluorescence results showed that the expression levels of MAP-2 in CUMS1 and CUMS2 rats were significantly lower than in the Control group, and also the vector and vehicle groups. From the histogram in Figure 6C [*F*_(7, 16)_ = 24.53, *P* < 0.0001], it can be seen that there is increasing expression in miR-16 and Fluoxetine groups (*P* = 0.0009 vs. CUMS1, *P* = 0.0398 vs. CUMS2) when compared to CUMS groups. While still less positive staining appeared in miR-16 and Fluoxetine groups (*P* = 0.0018 vs. Cont1, *P* = 0.0021 vs. Cont2) than in the control groups. NeuN expression levels from immunofluorescence among these groups can be seen in Figure 6A. And from the histogram in Figure 6D [*F*_(7, 16)_ = 26.53, *P* < 0.0001], it can be seen that it has similar tendencies to MAP-2. The expression of NeuN decreased after CUMS treatment (*P* = 0.0061 vs. Control), while miR-16 and Fluoxetine (*P* = 0.0005 vs. CUMS1, *P* = 0.0003 vs. CUMS2) can bring back expression toward the original level.

**Figure 6:** Immunofluorescence staining of NeuN and MAP-2 expression represent lower expressions of neuronal cells after CUMS. Expression levels of NeuN and MAP-2 are used to track neuron or dendrite formation. **(A)** Representative images of NeuN staining from each group. **(B)** Histogram of NeuN staining, a significant decrease presented in CUMS groups compared to the Control. Values are presented as means ± SEMs. ^*^P < 0.05; ^**^P < 0.001; ^***^P < 0.0001. **(C)** representative images of MAP-2 staining from each group. **(D)** Histogram from MAP-2 staining show similar change tendencies with NeuN expression in the rat hippocampus in each group. Values are presented as means ± SEMs. ^*^P < 0.05; ^**^P < 0.001; ^***^P < 0.0001.

### miR-16 and fluoxetine attenuated Bcl-2 down-regulation and Caspase-3 up-regulation induced by CUMS

As shown in Figure 7A, western blot analysis revealed changes in Bcl-2 and Caspase-3 expression levels. There were lower Bcl-2 expression in the CUMS1 and CUMS2 groups than in Cont1 and Cont2 group respectively. From the histogram in Figure 7B [*F*_(7, 16)_ = 117.1, *P* < 0.0001], the miR-16 group and the Fluoxetine treatment group were lower than controls (*P* = 0.0001 vs. Cont1, *P* = 0.0009 vs. Cont2) but higher than the two CUMS groups (*P* < 0.0001 vs. CUMS1, *P* = 0.0001 vs. CUMS2). Expression of Caspase-3 can be seen in Figures 7A,C [*F*_(7, 16)_ = 18.87, *P* < 0.0001], and when compared to the Cont1 and Cont2 groups, there was an increase in the CUMS1 and CUMS2 groups (*P* = 0.0016 vs. Cont1, *P* = 0.0423 vs. Cont2) respectively. Both miR-16 and Fluoxetine treatment groups (*P* = 0.0469 vs. CUMS1, *P* = 0.0298 vs. CUMS2) had the effect of attenuating this increase. Both the anti-apoptosis factor Bcl-2 and Caspase-3, which is a critical executioner of apoptosis, showed that CUMS could induce apoptosis. Moreover, the miR-16 group and Fluoxetine group reduced considerably the extent of this apoptosis.

**Figure 7:** Western blot was conducted to detect the expression level of Bcl-2 and Caspase-3 among each group. Western blot presents an increasing tendency in Bcl-2 in miR-16 and Fluoxetine treatment groups, but a decrease in CUMS groups, while an opposite change appears in Caspase-3 expression. **(A)** Compared with Control groups, the image shows a significant decrease in Bcl-2 expression in CUMS groups, but increasing Caspase-3 expression, and the miR-16 and Fluoxetine groups attenuate the change. The mean change in Bcl-2 **(B)** and Caspase-3 **(C)** are showed in the histogram. Values are the means ± SEMs. ^*^P < 0.05; ^**^P < 0.001; ^***^P < 0.0001.

### Beclin-1 and LC3II changes indicate that miR-16 and fluoxetine reduced CUMS induced autophagy

As is shown in Figure 8A, autophagic changes, represented by Beclin-1 and LC3II, were detected by western blot. From the histogram in Figure 8B [*F*_(7, 16)_ = 22.38, *P* < 0.0001], it can be seen that the gray value of Beclin-1 in CUMS1 and CUMS2 group (*P* = 0.0032 vs. Cont1, *P* = 0.0142 vs. Cont2) was significantly lower than the cont1 and cont2 groups, respectively. And this decreasing trend also appeared in the LC3II western blot results in Figure 8C [*F*_(7, 16)_ = 15.78, *P* < 0.0001]. However, when compared with CUMS1 and CUMS2 group (*P* = 0.004 vs. Cont1, *P* = 0.0336 vs. Cont2), the miR-16 group and Fluoxetine treatment groups had significant increases in both Beclin-1 (*P* = 0.0415 vs. CUMS1, *P* = 0.0045 vs. CUMS2) and LC3II (*P* = 0.0003 vs. CUMS1, *P* = 0.0291 vs. CUMS2) expression levels. When compared to CUMS1 and CUMS2 groups, the vector group and vehicle group had no such increase after CUMS (*P* > 0.05). The conclusion from these autophagic results is that CUMS induces a decrease in Beclin-1 and LC3II, but this is lessened with administration of miR-16 or Fluoxetine.

**Figure 8:** The expression levels of Beclin-1 and LC3II were detected by Western blot and revealed an autophagic decrease after CUMS. Western blot analysis of protein levels of Beclin-1 and LC3II in the rat hippocampus derived from each group. **(A)** The bands shown in the image presented a similar trend of Beclin-1 and LC3II expressions. Compared to the Control, the CUMS groups showed a significant decrease, while both miR-16 and Fluoxetine treatment bring back, to some extent, the change. Histograms from Beclin-1 protein levels **(B)** and LC3II **(C)** present the mean change, values are the means ± SEMs. ^*^P < 0.05; ^**^P < 0.001; ^***^P < 0.0001.

### Down-regulation of PI3K-AKT-mTOR detected by western blotting and immunofluorescence after CUMS

PI3K/Akt/mTOR pathways are widely considered to be one of the three major signaling pathways for cell survival and reproduction. From Figure 9C, western blot analysis revealed that CUMS treatment (*P* = 0.0027 vs. Cont1, *P* = 0.0003 vs. Cont2) decreased protein levels when compared with non-CUMS treated normal control rats. It can be seen from Figure 9D [*F*_(7, 16)_ = 23.28, *P* < 0.0001], Figure 9E [*F*_(7, 16)_ = 38.47, *P* < 0.0001], Figure 9F [*F*_(7, 16)_ = 124.5, *P* < 0.0001], that both miR-16 treatment and Fluoxetine treatment had the effect of significantly increasing of PI3K (*P* = 0.0381 vs. CUMS1, *P* = 0.0124 vs. CUMS2), Akt (*P* = 0.0474 vs. CUMS1, *P* = 0.0054 vs. CUMS2), and mTOR (*P* = 0.0098 vs. CUMS1, *P* = 0.0005 vs. CUMS2) expression compared to the CUMS1 and CUMS2 group respectively. From the images presented in Figure 9A [*F*_(7, 16)_ = 52.87, *P* < 0.0001, Figure 9B], it is clear that the CUMS groups had a significant decrease in the expression level of mTOR (*P* = 0.0018 vs. Cont1, *P* = 0.0012 vs. Cont2). However, miR-16 treatment and Fluoxetine treatment (*P* < 0.0001 vs. CUMS1, *P* = 0.0002 vs. CUMS2) was able to significantly increase PI3K/Akt/mTOR activity. Vector and vehicle groups did not show increased activity (*P* > 0.05) in PI3K, AKT or mTOR pathways in comparison with CUMS1 and CUMS2.

**Figure 9:** miR-16 treatment and Fluoxetine treatment was able to significantly increase PI3K/Akt/mTOR activity. **(A)** Images of mTOR Immunofluorescence staining show a decrease expression level in the CUMS groups compared with the Control groups. **(B)** Mean change in mTOR expression detected by immunofluorescence. **(C)** Compared with the Control groups, the protein expressions of mTOR, PI3K, and AKT levels decreased in the CUMS groups. Histograms from mTOR protein level **(D)**, AKT protein level **(E)** and PI3K protein level **(F)** show significant restoration toward control levels in both miR-16 and Fluoxetine groups. Values are the means ± SEMs. ^*^P < 0.05; ^**^P < 0.001; ^***^P < 0.0001.

## Discussion

In this paper we have shown that hsa-miR-16 can regulate Luciferase expression by targeting the 3′UTR portion of 5-HTT, hence confirming the regulatory binding site of miR-16 and 5HTT. A CUMS model was established and a miR-16 Lentivirus was injected to the rats' raphe nucleus, and its effect was assessed against that of Fluoxetine. Furthermore, detection of BDNF and 5-HT2a expression levels proved them to interact closely. Apoptosis and autophagic changes were also examined in relation to each group. Finally, we found the PI3K-AKT-mTOR regulatory pathway to be involved in the mechanism of both miR-16 and Fluoxetine.

SSRI are considered first line in pharmacologic treatment for patients with MDD. However, despite rapidly penetrating certain areas of the brain, they have a delayed onset of action. In our study, drugs were not administered until our depression model had been proved to be successful with behavioral testing. Thus treatment was given post stress to animals still suffering from depression. Treatment post diagnosis of depression is reflective of what happens in a clinical setting. Furthermore, it is in accordance with procedures in previous studies (Hirano et al., 2005). It is possible that if the time gap between stressing ending and animal testing starting is not sufficient, the changes could not be caused only by depression, but also by the physiological reaction to recent stress. If this is the case, the effect on test results would be equal on all stressed experiment groups. Also, if testing results were affected by the fact that changes were due to a combination of depression and the physiological response to a recent stressing, and not purely depression, the changes would most likely become more or less pronounced over the course of the experiment as the contributing levels of depression increased over time while the effect of the recent stressing would remain more constant, because the time gap was kept constant. An equal time interval was used. Therefore, it is possible that results were not solely due to depression, but we did not prove or disprove this in this paper. Increasing evidences have demonstrated reduced 5-HT neurotransmission as a primary defect in depression and the SSRI has been used as the most effective treatment for depression. The SSRI could be effective since serotonin transporter (SERT) ensures the recapture of serotonin thus conduct pharmacologicaltarget effects. Furthermore, it has been identified that the SERT-targeting miRNA miR-16 could be involved in relaying SSRI anti-depressant action. Also increased cortical 5-HT2a receptors have been widely quoted to be associated with depression-related personality characters.

Pierre Blier has suggested two of the chief effects of SSRIs are enhancing synaptic levels of 5-HT and decreasing the firing activity of NE and DA neurons (Blier, 2016). Traditionally, it has been widely accepted that blockade of the 5-HT2A/2C receptor can improve learning (Meneses, 1999). Albert et al. suggested modifying 5-HT1A receptor gene expression as a new approach to antidepressant therapy (Albert and Francois, 2010), and another research indicated DNA methylation as one method of modifying the 5-HT1A receptor (Le Francois et al., 2015). In addition, 5-HT2AR-D2R functional crosstalk has been discovered to provide a novel angle for signal integration between the serotonin and dopamine systems (Albizu et al., 2011). Moreover, it has been found that antidepressant therapy can be beneficially conducted via a single cell type in the cerebral cortex, and targeting CStr neurons has potential for developing drugs (Schmidt et al., 2012). In this study, 5-HT2a expression levels were compared between control rats and CUMS rats, and was consistent with previous research where mice subjected to chronic stress had increased 5-HT 2AR (Tianzhu et al., 2014). Recently, it has been suggested that 5 HT2AR concentration in platelet lysate is involved the pathology of depression (Liu et al., 2015) and 5-HT2a could contribute to altered systemic lipid- and glucose metabolism (Hansson et al., 2016). In accordance with a study that revealed 5-HT2A receptor antagonist treatment being able to reverse depressive-like behaviors (Xu et al., 2016), our results showed that both miR-16 and Fluoxetine treatments can decrease 5-HT2A levels and attenuate depressive behavior in rats.

The role of microRNA has been studied in many diseases during recent years. Several previous studies have demonstrated that miR-16 plays a role in the therapeutic action of SSRI antidepressants in monoaminergic neurons (Baudry et al., 2010) and it has been hypothesized that SSRI antidepressants conduct promotion of neurogenesis by regulating bcl-2 levels through miR-16 in the hippocampus (Launay et al., 2011). Moreover, it has been discovered that miR-16 up-regulation and BNDF down-regulation play a role in the development of depression-like behaviors in the hippocampus (Bai et al., 2012) and miR-16 can also regulate multiple serotonergic pathway-related genes (Moya et al., 2013). According to previous studies, there was a decrease of CSF miR-16 in MDD but an increase of serum miR-16 after CUMS (Song et al., 2015; Zurawek et al., 2016). This study injected miR-16 into the raphe nucleus and observed a significant attenuation of depressive like behaviors, in fact as effective as Fluoxetine treatment. For human studies, miR-16 has been suggested to be a biomarker of anxiety (Honda et al., 2013). O'Conner et al. proposed that many miRNAs can increase the complexity of their regulatory capacity by binding to the 5′UTR of mRNAs and it may be possible to produce a more robust and rapid anti-depressive effect with less side effects by directly controlling related targeting miRNAs (O'Connor et al., 2012, 2013). Other microRNAs to have been reported to be related to depression are miR-34 acting as a regulator of CRF signaling, miR-134 and miR-124a levels were significantly downregulated after treatment with duloxetine and miR-144 was found to have an increased expression in both lithium- and valproate-treated animals (Haramati et al., 2011; Hansen and Obrietan, 2013; Pan and Liu, 2015). In addition, overexpression of miR-135a in 5HT Neurons was proved to reduce depression-like behaviors (Heyer and Kenny, 2014; Issler et al., 2014).

Apoptosis and autophagy are two degradation processes, which are pivotal in response to stressed related conditions. It has been demonstrated that hippocampal newborn cell deficiency was observed after CMS and was involved not only in apoptosis, but also in impairing novel circuit establishment (Wang et al., 2012). In this present study, Bcl-2 and Caspase-3 downregulation were examined, which indicated that anti-apoptosis status is reduced after CUMS, but can be brought back to some extent by both Fluoxetine treatment and miR-16 injection. Apoptosis process regulation is very closely related to the autophagic process. Beclin-1 (the mammalian orthologue of the yeast autophagy protein Apg6/Vps30) is one of the critical proteins during this process, together with autophagic marker LC3 II, so these were detected by western blotting in this study. The results showed a decrease after CUMS when compared to controls, however this was reversed by antidepressant treatments. These results were in accordance with previous reports that the abundance of autophagic markers rises with antidepressant treatment *in vitro* (Gassen et al., 2015). PI3K-AKT-mTOR is generally considered to regulate survival through proapoptotic inhibition or anti-apoptotic activation. Previous study has revealed that autophagy contributes to synaptic plasticity and other brain functions through PI3K–Akt–mTOR pathway inhibition (Shehata et al., 2012). Another study found that creatine and ketamine can reverse depressive-like behavior and the underlying mechanism is through regulation of the PI3K/AKT/mTOR pathway, and modulation of synaptic proteins and BDNF in the hippocampus (Pazini et al., 2015). Currently, it has been discovered that stressful events could affect BDNF expression level in hippocampal thus induce depressive phenotypes. While the underlying mechanisms regulate BDNF expression remain unclear. Recently, miR-16 has been identified to be involved in SRI antidepressant action in serotonergic raphe by mediating adult neurogenesis in the mouse hippocampus. Generally, the effect of miRNA rely on its translational repression on mRNA expression through binding the 3′UTR (3′ untranslated region). It has been uncovered by bioinformatics target analysis that potential regulatory of miR-16 was identified to be a candidate miRNAs for the BDNF gene. In our study, miR-16 and BDNF expression levels were detected by RT PCR, and showed a significant decrease in BDNF after CUMS. Also, MAP-2 and NeuN expression were assayed by immunofluorescence and showed a decrease in neuronal cells. Decreased dendritic spine density and dendritic branching is associated with psychiatric disorders (Xu et al., 2016). It has been reported that alleviation of depressive-like behavior can be traced to increasing expressions of BDNF and p-TrkB (Lin et al., 2016; Su et al., 2016).

A decade ago, it had been already been pointed out that epidemiologically 40–50% of the risk in depression is genetic and therefore a wise direction for future study would be to identify specific variations that both confer or resist depression (Nestler et al., 2002). Consequently, many researches took this approach, for instance, the Tph2 gene has been proposed as a causal factor in 5-HT deficiency both clinically and preclinically (Jacobsen et al., 2012). Besides, some epidemiological evidence indicated a neuroendocrine link between stress, depression and diabetes, subsequently a study discovered that glucose intolerance and its associated increased risk of diabetes in CUMS rats resulted from the loss of insulin signaling (Pan et al., 2013). In addition, new molecular strategies have come to the forefront of current research. For example, silencing specific target genes by RNA interference (RNAi) strategies have been used to evoke antidepressant-like effects in laboratory animals by knocking down the expression of the serotonin transporter (SERT) or the 5-HT1A auto receptor (Bortolozzi et al., 2014). Future studies would be to further explore miR-16 or Fluoxetine treatment to autophagic flux changes during depression development and how these changes related to the apoptosis process, neurotransmitters and the relevant receptors. And such research may well provide the basis for clinical treatment of depression with a shorter response time, a higher efficacy and less severe side effects.

## Author contributions

MF designed the experiments and YY drafted the manuscript; YY, XD, and ZH participated in the study design and coordination; YY and XD performed the experiments; YY, XH, and ZH analyzed the data and HD revised the manuscript. All authors read and approved the final manuscript.

### Conflict of interest statement

The authors declare that the research was conducted in the absence of any commercial or financial relationships that could be construed as a potential conflict of interest.

## Supplementary material

Supplementary Figure 1 Merged immunofluorescence images of representative slices from the raphe nuclei. Merged images of anatomical representation of physical locations of the sites of injection, the nuclei were stained by DAPI, blue channel. The expression of GFP, green channel **(A,B)**. Rat brain atlas, raphe nuclei marked as red **(C)**.

## Abbreviations

SSRI: Selective Serotonin Reuptake Inhibitor
CUMS: Chronic Unpredicted Mild Stress
SERT: Serotonin Transporter
MDD: Major Depressive Disorder
CNS: Central Nervous System
miRNA: Micro ribonucleic acid
PI3K: Class III phosphatidylinositol kinase
BDNF: Brain Derived Neurotrophic Factor
PVDF: Polyvinylidine difluoride
5-HT: 5-hydroxytryptamine
AKT: Serine/threonine Kinase
mTOR: Mammalian target of rapamycin.
